# Pathogenesis, clinical manifestations and complications of coronavirus disease 2019 (COVID-19)

**DOI:** 10.2217/fmb-2020-0110

**Published:** 2020-08-27

**Authors:** Elaheh Kordzadeh-Kermani, Hossein Khalili, Iman Karimzadeh

**Affiliations:** ^1^Department of Clinical Pharmacy, Faculty of Pharmacy, Tehran University of Medical Sciences, Tehran 141761441, Iran; ^2^Department of Clinical Pharmacy, Faculty of Pharmacy, Shiraz University of Medical Sciences, Shiraz 7146864685, Iran

**Keywords:** clinical complications, coronavirus disease 2019, pathogenesis, SARS-CoV-2

## Abstract

**Aim:** Despite the similarities in the pathogenesis of the beta coronaviruses, the precise infective mechanisms of SARS-CoV-2 remain unclear. **Objective:** In this review, we aim to focus on the proposed theories behind the pathogenesis of SARS-CoV-2 and highlight the clinical complications related to coronavirus disease 2019 (COVID-19). **Methods:** We conducted a literature search in Pubmed, Scopus and Google Scholar for the relevant articles regarding clinical complications and pathogenesis of COVID-19. **Results:** Related articles were included and discussed. **Conclusion:** Respiratory system and the lungs are the most commonly involved sites of COVID-19 infection. Cardiovascular, liver, kidneys, gastrointestinal and central nervous systems are involved with different frequencies and degrees of severity.

In December 2019, a novel coronavirus (initially named 2019-nCov) was discovered to be responsible for the outbreak of unusual series of viral pneumonia of unknown origin in Wuhan, Hubei province of central China. 2019-nCov was later named SARS-CoV-2, because of the structural similarities with the SARS-CoV, which caused the outbreak of SARS in 2003 [1]. The number of infected cases outside China exponentially increased across the continents. As of 22 July 2020, over 14.9 million confirmed cases and more than 610,000 deaths related to COVID-19 have been reported worldwide, raising a global concern [2]. SARS-CoV-2 is an enveloped, single-stranded ribonucleic acid betacoronavirus. This highly contagious pathogen is transmitted by respiratory droplets and aerosols, direct contact of mucous membranes and probably the fecal–oral route [3] As described by the Centers for Disease Control (CDC), the most common symptoms of the illness include fever, cough, fatigue, anorexia, dyspnea, sputum production and myalgia [4,5], however, a significant number of infected cases (43.8%) do not exhibit fever or radiological abnormalities on the initial presentation [5]. Therefore, human-to-human transmissions are facilitated by unidentified asymptomatic carriers (particularly healthcare providers) during the incubation period (usually 5–7 and as long as 28 days) [6].

The actual mortality rate of SARS-CoV-2 infection is ill defined and significantly differs around the world, ranging from 0.3–8.4%. Tang *et al.* discovered two major types of SARS-CoV2 from 103 human samples; the L type, which is presumed to be more aggressive, and the S type, which is probably evolved from the L type with less aggressive features. It is not clear if these relatively small mutations have impacts on the virus pathogenesis and the wide range of mortality [7]. Ellinghaus *et al.* recently found a connection between chromosome 3p21.31 and the severity of COVID-19. The authors also presumed that individuals with blood group A are more likely to develop severe disease [8].

Since the outbreak of COVID-19, extensive attention has raised to combat the spread of the virus. To date, no therapeutics has been established to be effective against COVID-19. Despite the lack of evidence from clinical trials, chloroquine and hydroxychloroquine were authorized by the US FDA to be used in COVID-19 based on the *in vitro* studies and a small nonrandomized clinical trial. Laboratory data suggested that these antimalarial drugs could interact with the ACE 2 receptors, increase the pH of the host cell and inhibit viral endocytosis [9]. A growing body of evidence suggests that chloroquine and hydroxychloroquine are probably not effective against COVID-19 [10], and concerns about their cardiovascular toxicity, especially in severe COVID-19, restrict their use. Based on the recent evidence, the WHO temporarily suspended the hydroxychloroquine safety trial in May 2020. Remdesivir is an antiviral agent that demonstrates *in vitro* activity against SARS-CoV-2 via inhibiting the RNA polymerase. It has been authorized by the FDA to be used in severe COVID-19. The clinical efficacy of remdesivir against COVID-19 is controversial. Randomized clinical trials have demonstrated the possible benefit of remdesivir in reducing the time to recovery in severe COVID-19 infection [11,12]. However, remdesivir has not been found to reduce the viral load in nasopharyngeal swabs of the treated patients [12]. In a recently published cohort of 62 severe COVID-19 patients, clinical improvement was observed in 36 of the cases. Nevertheless, the results of this study could be affected by the small sample size, lack of randomization and short duration of follow-up [13].

Scientists have been making a lot of effort to discover a protective vaccine against SARS-CoV-2. Chinese experts have evaluated the tolerability and immunogenicity of adenovirus type-5 vectored COVID-19 vaccine within 28 days of vaccination in 108 participants. Humoral response to the vaccine was observed on day 28 of immunization [14]. In USA, preliminary results of the mRNA-1273 vaccine were successful and it is currently in Phase II for evaluation [15]. On the other side of the world, researchers of Oxford University are recruiting for Phase II/III of the COVID-19 vaccine (ChAdOx1) [16].

Several theories have been made to explain the pathogenesis behind the complications of and death due to COVID-19 [17–25]. This study aims to critically review the published literature on clinical characteristics, laboratory abnormalities and histopathological findings of COVID-19 infection. We also discuss expert opinions regarding the pathogenic mechanisms causing clinical symptoms and complications of COVID-19 as well as the contributing factors leading to organ dysfunction. Acknowledgment of the underlying pathophysiology provides new perspectives in the management of the infection. It can also help researchers to design and offer more effective and targeted options for the treatment of COVID-19.

## Methods

We conducted a literature search in Pubmed, Scopus and Google Scholar for the relevant articles regarding clinical complications and pathogenesis of COVID-19 from January 2020 up to 15 June 2020. We used search terms related to each of the human organs, and clinical complications along with ‘COVID-19’, ‘Coronavirus’, ‘2019 novel coronavirus’, ‘2019-nCov’ and ‘SARS-CoV-2’. Research articles, review papers, research letters, case reports and commentaries were included. The articles closely related to our study were discussed in this review.

## Pathogenesis

Following viral transmission, SARS-CoV-2 attaches to the surface of the epithelial membrane of the oral cavity, the mucosal membranes of the conjunctiva or the otic canal. Angiotensin-converting enzyme 2 (ACE 2) protein, which is highly expressed on multiple human cells including type II alveolar cells (AT2), oral, esophageal, ileal epithelial cells, myocardial cells, proximal tubule cells of the kidneys as well as urothelial cells of the bladder [17] is believed to mediate the internalization of SARS-CoV2. The spike (S) protein of SARS-CoV2 is cleaved by a cellular enzyme named furin at the S1/S2 site. This cleavage is essential for viral entry to the lung cells [26]. The activated S protein is primed by the *Tansmembrane Serine Protease 2* *(TMPRSS2)* and finally attaches ACE 2 receptors to enter the host cells. The genetic sequence of SARS-CoV-2 is homologous with the SARS-CoV, and the structure of (S) protein of these viruses is highly similar. They both use the same receptor to enter the host cell; however, SARS-CoV-2 binds ACE 2 receptors with tenfold higher affinity [18].

Experimental studies suggest that the ACE 2/angiotensin (1–7) has a fundamental role in inflammation and signaling pathways contributing to tissue injury [27]. The physiological role of ACE 2 is the degradation of angiotensin II and the production of angiotensin (1–7), which counteracts ACE II [19]. Following the viral replication in the host cell, downregulation of ACE 2 inhibits breakdown of angiotensin II into angiotensin (1–7). Disturbance in ACE 2/angiotensin (1–7) axis explains particular clinical features of COVID-19, such as hypokalemia, vasoconstriction [28] and development of acute respiratory distress syndrome (ARDS) [20]. Interestingly, the extent of ACE 2 expression in the gastrointestinal (GI), cardiovascular, genitourinary, endocrine (pancreas) and genitourinary (testis) systems is extremely higher than that in the predominant target of the virus, the respiratory system [17]. Evidence has not shown the presence of SARS-CoV-2 in some organs enriched with ACE 2 receptors, such as expressed prostatic secretion of COVID-19 patients [21]. Hence, there is no correlation between the virus infectivity and the level of ACE 2 expression. Limited evidence suggests that ACE 2 expression is attenuated in females compared with the males which could justify the higher number of COVID-19 cases in men [29,30]. Besides, investigators in the Mount Sinai Health System, New York, have found that the expression of ACE 2 is age dependent [31].

Wang *et al.* identified CD 147 receptors as a novel route for the invasion of the virus. They showed that anti-CD147 humanized antibody inhibits the viral entry to host cells [22]. It is not definite if the virus invades the host cells using alternative mediators.

The severity of COVID-19 is positively correlated to the level of inflammatory cytokines such as interleukins (IL-2, IL-6, IL-7, IL-10), granulocyte colony-stimulating factor (GCSF), interferon gamma-induced protein 10 (IP-10), monocyte chemoattractant protein-1 (MCP-1), macrophage inflammatory protein 1 alpha (MIP-1A) and tumor necrosis factor -alpha (TNF-α). In patients with severe disease, a significant reduction in lymphocyte count is observed [24,25,32]. Flow cytometric analysis of severe COVID-19 patients demonstrates a remarkable reduction of lymphocytic T Cells (CD4^+^ and CD8^+^) and natural killer (NK) cells. Besides, an increase in the expression of natural killer group 2 A (NKG2A), programmed cell death protein 1 (PD-1) and T-cell immunoglobulin mucin-3 (Tim-3) is associated with functional exhaustion of T lymphocytes in the early stage of the disease [24,25]. NKG2A is an inhibitory member of the NKG2 family and is expressed on NK cells, natural killer T (NKT) cells and a subset of CD8^+^ T cells. Interaction of NKG2A with histocompatibility antigen alpha chain E (HLA-E) can inhibit the activation of NK cells, and T cells [33]. PD-1 is expressed on both the T lymphocytes and NK cells. It is involved in subsiding immune responses and promoting self-tolerance through suppressing the activity of T cells and promoting differentiation of regulatory T cells [34]. T-cell immunoglobulin mucin-3 (Tim-3) is a co-inhibitory receptor that is expressed on IFN-γ producing T cells, and innate immune cells (e.g., macrophages and dendritic cells). It plays a key role in inhibiting T helper 1 cells (Th1) responses and the expression of cytokines such as TNF-α and IFN-γ [35].

## Clinical manifestations

People of all ages are susceptible to COVID-19 infection. Children and adolescents under 18 years represent under 2% of the confirmed COVID-19 cases [36]. Several studies indicate that the majority of the infected children are asymptomatic or experience mild symptoms during the COVID-19 pandemic [37]. Of the infected children, 11% require hospitalization. Most children survive the disease and death related to COVID-19 is uncommon in cases aged under 18. In a cohort of 100 children admitted in the emergency in Italy low-grade fever (54%), cough (44%) and anorexia (23%) were observed. Severe disease was observed in 1–2% of the cases [38].

The common clinical features of COVID-19 pneumonia in adults include fever, dry cough, sore throat, headache, fatigue, myalgia and breathlessness [39,40]. The disease manifestations in the infected patients range from mild pneumonia (81%) to moderate pneumonia (hypoxia requiring hospitalization, 14%), and critical illness (leading to invasive mechanical ventilation, multiorgan dysfunction and possibly death, 5%). The risk of death depends on age, underlying comorbidities and severity of the disease, increasing up to 49% in critically ill patients [41]. Epidemiologic data from China indicate that independent of age, men are at greater risk for the development of severe COVID-19 compared with women [42]. Underlying comorbidities including cardiovascular disease, chronic kidney disease, chronic lung disease, diabetes and malignancy are associated with increased risk of severity of COVID-19 [41]. Obese patients as defined by BMI of at least 30 Kg/m^2^ are at greater risk of deterioration of the disease and requirement of intensive care unit (ICU) care [43] Zhou *et al.* reported that older age (odds ratio 1·10, 95% CI: 1·03–1·17, per year increase; p = 0.0043), higher sequential organ failure assessment (SOFA) score (5·65, 2·61–12·23; p < 0.0001), and D-dimer of greater than 1 μg/ml on admission (18·42, 2·64–128·55; p = 0.0033) were significantly associated with the mortality of adult inpatients with COVID-19 in Wuhan, China. Recovery was observed in the second or third week from symptom onset. The median duration of hospitalization in individuals who recovered was 10 days. The most affected organs were the lungs, followed by the heart, kidneys, liver, brain and gastrointestinal system [44].

According to data obtained from a series of rheumatoid arthritis patients on immunosuppressive therapies, the clinical course of COVID-19 does not seem to be significantly affected by the biological disease-modifying antirheumatic drugs (bDMARDs) or targeted synthetic disease-modifying antirheumatic drugs (tsDMARDs) [45]. As opposed to the rheumatoid arthritis population, recipients of organ transplant are at a very high risk of death related to COVID-19; 28% of the cases of kidney transplant at Montefiore Medical Center, New York City, died due to COVID-19 [46].

## Complications

### Respiratory system involvement

The predominant manifestation of COVID-19 is the involvement of the respiratory system presenting as interstitial and alveolar pneumonia. Thin slice chest computerized tomography (CT) is useful for early detection of COVID-19 pneumonia. The CT scan of COVID-19 patients demonstrates a various pattern, ranging from single ground-glass opacity (GGO) to bilateral diffuse heterogeneous consolidation with air bronchogram and bronchiectasis, the ‘white lung’. The typical radiological pattern in the early phase of the disease is GGO predominantly distributed in the peripheral subpleural areas of the right lower lobes, which later develops into GGO with inter or/and intralobular septal thickening as crazy-paving pattern. As the disease progress, a CT scan demonstrates subsegmental and bilateral multiple lobular consolidations. Minimal pleural effusion, lymphadenopathy, the reversed halo sign and pulmonary nodules are infrequently reported in COVID-19 pneumonia [47,48].

The mortality rate of COVID-19 increases by up to 49% in patients who develop ARDS. Age, neutrophilia, elevated LDH and D-dimer are the identified risk factors for the development of ARDS [51]. Similar to the MERS, a positive association of neutrophilia and lung damage has been recognized in COVID-19 [49]. In the histopathological analysis of the lungs of severe COVID-19 patients, pathological patterns of ARDS similar to SARS (diffuse alveolar damage, desquamation of pneumocytes, development of hyaline membranes, edema and interstitial infiltrations) have been observed. The virus cytopathic effect is suggestive of the direct invasion of SARS-CoV-2 to pneumocytes [50,51]. In a report of the autopsies from four decedents, accomplished in New Orleans, lymphocytic infiltrations (CD4^+^ and CD8^+^) accompanied by platelet-rich thromboses were observed [52].

Invasion of SARS-CoV-2 to pneumocytes results in reduced expression of ACE 2 and cleavage of angiotensin II to develop angiotensin (1–7). Angiotensin (1–7) has a fundamental role in protecting the lungs from deterioration to ARDS. By contrast, intact angiotensin II stimulates pro-inflammatory responses and increases vascular permeability of the lung tissue, which leads to ARDS [53]. The role of T cell lymphocytes, neutrophils and macrophages in COVID-19 has not been completely understood. Flow cytometric analysis of critically ill COVID-19-infected patients demonstrated that significant lung injury is accompanied by a substantial decrease in the number of CD4^+^, CD8^+^ T lymphocytes and NK cells. Elevated IL-6, increased Th 17 in CD4^+^ T lymphocytes and cytotoxicity of CD8^+^ T cells are speculated to stimulate the immune response and induce cytokine release syndrome (CRS), which finally results in ARDS and multiorgan failure [54].

### Cardiovascular involvement

Hypertension, diabetes, heart failure and coronary artery disease are the most particular comorbidities that have been identified in COVID-19 patients. Imbalanced activation of the ACE 2/angiotensin (1–7) pathway is associated with a pro-inflammatory state and is assumed to cause more severe disease in patients with cardiovascular comorbidities. Besides, treatment with ACE inhibitors/angiotensin II receptor blockers (ARB) and high level of ACE 2 expression could result in delayed viral clearance and propensity of these individuals to COVID-19 [55,56]. Conflicting theories have been made regarding the implications of renin-angiotensin system (RAS) inhibitors on the propensity to COVID-19 infection [57]. Some experts are concerned about the theory that upregulated ACE 2 receptors may be associated with increased SARS-CoV-2 infectivity. On the contrary, others contemplate that ACE inhibitors/angiotensin 2 receptor blockers (ARBs) may decrease the severity of COVID-19 and have beneficial effects [58]. Because of the potential harm of discontinuation of ACE inhibitors and ARBs and lack of prospective clinical evidence, the international societies recommend continuing these medications in COVID-19 patients as well as the uninfected ones [56].

The mortality rate of COVID-19 is estimated at over 10% in patients with low cardiac reserve (heart failure and coronary artery disease). Elevated hs-Troponin I and electrocardiogram (ECG) abnormalities, as indicative of myocardial injury, were detected in 7.2% of the patients admitted in a hospital in Wuhan; with the advancement of the disease in 22% of the cases, critical care was required [39]. The pathophysiologic reason to explain the mortality of COVID-19 in cardiovascular diseases was recently explained by Xiong *et al.* Myocyte injury occurs when metabolic demands induced by viral inflammation increase the challenge for a weak heart [59]. Neither direct viral invasion of the virus to heart tissue nor lymphocytic infiltration consistent with myocarditis has been reported from the pathological analysis [50]. Remarkably, myocyte necrosis was observed in autopsy analysis of patients from New Orleans, which suggests that SARS-CoV-2 could invade the pericytes and cause micro-circulation dysfunction [50,59,60].

In a case series in Evergreen Hospital, Kirkland, Washington, cardiomyopathy developed in 8 of the 21 (38.09%) COVID-19 patients admitted to ICU [61]. Cardiomyopathy is assumed to be a late complication of severe COVID-19; meanwhile, in few case reports, myocarditis was observed as a primary manifestation [62–64]. In one case report, viral myocarditis associated with COVID-19 occurred without any sign and symptoms of pneumonia [65]. In another report, cardiac tamponade associated with COVID-19 in a 47-years-old female with no underlying risk factors was surprisingly described [66]. The invasion of the viruses in the bloodstream mediated by ACE 2 receptors highly distributed in the heart and endovascular system stimulates CRS. Myocyte apoptosis could occur as a consequence of subsequent infiltration of neutrophils, and imbalanced T helper response [67]. It is presumed that immune-mediated response is the main pathogenic mechanism in cardiomyopathy related to COVID-19. Therefore, in the treatment of the reported cases, immunomodulatory agents such as hydrocortisone, methylprednisolone, intravenous immunoglobulin (IVIG), tocilizumab and hydroxychloroquine have been used [62,63,68,69].

In the Chinese study in Wuhan, of the 36 patients who were transferred to the ICU, arrhythmia was observed in 16 (44%) individuals [39]. Increased sympathetic nervous system activity due to myocarditis and pro-inflammatory state are contributing factors to the development of cardiac rhythm abnormalities [67]. Apart from these factors, hypoxia, hypotension, ACE 2-receptors downregulation, drug toxicity/interaction could also lead to developing or aggravating arrhythmic complications in patients with COVID-19 [70].

Therefore, cardiac monitoring, electrolyte balance (particularly potassium maintenance due to urinary potassium loss) and management of drug interactions with particular attention to arrhythmogenicity (e.g., chloroquine, hydroxychloroquine, lopinavir/ritonavir), rational use of fluid should be considered to decrease the fatality rate. Patients with cardiovascular diseases should be strongly advised to adhere to current ACC/AHA guidelines on pneumococcal and influenza vaccination [71]. To decrease the mortality rate of individuals with underlying cardiovascular comorbidities, effective metabolic control (blood glucose, lipid profile and blood pressure) is strongly advised [53].

### Kidney involvement

Acute kidney injury (AKI) is one of the major contributing factors of COVID-19-related death [72]. Similar to SARS-CoV and MERS, the kidneys are potential targets for COVID-19 [73,74]. Podocytes and proximal tubular epithelial cells highly enriched with ACE 2 receptors, are distinctive targets for SARS-CoV-2 [75]. In a multi-centered, retrospective, observational study in two hospitals in Wuhan, China, more than a fourth (28%) of the cohort developed AKI. Proteinuria, hematuria, increased levels of blood urea nitrogen and serum creatinine were present in 59, 44, 14 and 10% of patients, respectively. These variables, along with urine analysis and D-dimer, were significantly associated with the death of COVID-19 patients [76]. The existence of microalbumin, α1-microglobulin, immunoglobulin-G and transferrin in urine analysis of 12 patients confirms glomerular and tubular injury associated with COVID-19 infection [77]. A recent systematic review and meta-analysis have reported that the overall incidence of AKI in all COVID-19 patients was 4.5%. In mild or moderate cases, severe cases and critical cases of COVID-19, the incidence of AKI was 1.3% (95% CI: 0.2–2.4%), 2.8% (95% CI: 1.4–4.2%) and 36.4% (95% CI: 14.6–58.3%), respectively. On the other hand, the incidence of AKI was 52.9% (95% CI: 34.5–71.4%) and 0.7% (95% CI: -0.3 to 1.8%) in nonsurvivors and survivors, respectively. Therefore, AKI appears to be closely associated with both the severity and prognosis of COVID-19 patients [78].

Diao *et al.* recently described the pathophysiology of AKI associated with COVID-19. Histopathological analysis from autopsies of renal tissue of COVID-19 patients demonstrates that SARS-CoV-2 directly targets the renal tubules (enriched with ACE 2 receptors) via the systemic circulation. Subsequently, complement-mediated response and infiltration of CD68^+^ macrophages to the tubulointerstitial tissue cause further damage and fibrosis [73]. Dehydration, the use of nephrotoxic medications such as nonsteroidal anti-inflammatory drugs (NSAIDs), diuretics, ganciclovir and vancomycin, rhabdomyolysis, hypoxia, shock and underlying diseases (uncontrolled diabetes or hypertension) are other possible mechanisms which could be attributed to AKI during hospitalization [72].

Monitoring of kidney function, rational fluid administration, maintaining electrolyte and acid-base balance, avoidance of unnecessary nephrotoxic drugs, appropriate drug dosing and considering renal support via hemodialysis or continuous renal replacement therapy (CRRT) in advanced kidney injury is of significant importance to improve survival [72,75].

### Hematologic involvement

Thrombocytopenia associated with COVID-19 reflects the severity of the disease [79]. Coronavirus may invade the hematopoietic cells or cause abnormal hematopoiesis secondary to immune system response [80]. In addition, virus-induced alveolar damage affects the resident megakaryocytes in the lungs (decrease platelet production). The presence of active CD61^+^ megakaryocytes in autopsy examinations of the lungs confirms this theory [52]. Finally, endothelial damage related to coronavirus infection and mechanical ventilation could lead to platelet aggregation as well as thrombus formation (increased platelet consumption) [79,81].

In post-mortem inspection of six patients infected with COVID-19, evidence of viral damage to the spleen and lymph nodes (congestion, hemorrhage, atrophy, depletion of lymphoid follicles) has also been observed. Immunofluorescence staining of the spleens has shown that SARS-CoV-2 targets CD169^+^ macrophages and lymphocytes. Apoptosis may occur as a result of cytokine production (IL-6), predominantly secreted by the infected CD169^+^ macrophages [82].

### Coagulopathy

Histopathological evidence confirms the existence of thrombosis in pulmonary vessels in severe COVID-19 [52]. In a retrospective study on 183 COVID-19 patients in Wuhan, China, 15 (1.4%) and one (0.6%) of the nonsurvivors and survivors had overt disseminated intravascular coagulation (DIC), respectively. The median time from hospital admission to DIC development was 4 days (range, 1–12 days) [83]. Markedly elevated D-dimer and fibrin degradation products (FDP) (indicators of thrombin generation), along with thrombocytopenia in the latest stage of severe COVID-19 is implicative of hyperfibrinolysis and occurrence of sepsis-induced coagulopathy (SIC) [83]. Based on the results from the analysis of the observational studies, D-dimer and FDP elevations, are independent risk factors for mortality and could be useful for the early identification of severe disease [84]. The International Society of Thrombosis and Hemostasis (ISTH) recommends a risk stratification tool to make decisions on patient admission using D-dimer level, prothrombin time (PT) and platelet count [85]. Of note, the prophylactic dose of low molecular heparin (LMWH) has been demonstrated to improve the outcome of patients with sepsis-induced coagulopathy (SIC) score ≥4 or D-dimer >3.0 μg/ml (>6 upper limit of normal) [86]. Low dose unfractionated heparin (UFH) could be considered if overt thrombosis associated with DIC occurs [87]. Ji *et al.* highlighted the possible role of plasmin in increased pathogenicity of the virus. Plasmin cleaves the S protein of the virus and probably increases its affinity to attach ACE 2 and enhance viral entry into the host cells. Elevated plasmin activity is a common feature of COVID-19 patients with underlying comorbidities (hypertension, diabetes, heart failure); and could justify the increased risk of mortality rate in these patients [88].

Severe COVID-19 patients are at increased risk of thrombosis due to immobility, inflammatory state, hypoxia-induced thrombosis and potential invasion of the virus to endothelial cells. Endothelial cells are potential targets for the SARS-CoV-2 because of the highly expressed ACE 2 receptors. Endothelial damage and impairment of the natural anti-inflammatory state are likely to be associated with COVID-19 related coagulopathy [89]. Ranucci *et al.* investigated the procoagulant pattern of COVID-19 patients complicated by ARDS; according to a logarithmic regression represented by the authors, fibrinogen levels correlate with IL-6 levels. This finding is indicative of the link between the proinflammatory state and coagulopathy of COVID-19 [90]. The presence of antiphospholipid antibodies accompanied by cerebral infarcts has been reported in a few cases of critically ill COVID-19 patients. In all three of the cases, patients had underlying comorbidities, particularly hypertension. It is unclear if COVID-19 stimulates the production of antiphospholipid antibodies [91].

### Electrolyte imbalance

The impact of SARS-CoV-2 on the ACE-Ang II system leads to the inhibition of Ang II degradation. Intact Ang II promotes aldosterone production and enhances urinary potassium loss [20,55]. Moreover, in patients with severe diarrhea and/or vomiting, extrarenal potassium loss could also cause or aggravate hypokalemia. Hypokalemia is a known risk factor associated with exacerbation of ARDS and arrhythmogenicity.

Hypophosphatemia has been observed to correlate with lymphocyte count and severity of COVID-19. In a small study in China of 20 critically ill patients, hypophosphatemia was observed in 50% of the severe cases. The stress burden of the viral infection and gastrointestinal losses due to impairment of the mucosal integrity could contribute to hypophosphatemia. Maintenance of the serum phosphorus level within the normal range may improve respiratory support and promote the function of the immune system [92].

A literature review by Lippi *et al.* on five studies demonstrated that electrolyte imbalances, including lower serum concentrations of sodium, potassium and calcium, have been observed in patients with severe COVID-19. However, the precise mechanisms and clinical relevance of these electrolyte abnormalities are not completely understood [93].

### Liver involvement

The Pooled analysis of the 243 patients from eight studies suggests that AST elevation occurs in 20% of the COVID-19 patients (95% CI: 15.3–25.6%). Data pooled from six studies including 197 patients indicates that ALT elevation is observed in 14.6% of COVID-19 cases (95% CI: 12.8%–16.6%) [94]. Other reports indicate that in 14–53% of COVID-19 cases, abnormal levels of aminotransferases (AST and ALT) are observed [95]. Gamma-glutamyltransferase (γ-GT) and lactate dehydrogenase (LDH) has also been found to be elevated in 44.4 and 31.58% of COVID-19 cases, respectively [96]. Elevated alkaline phosphatase (ALP) level was observed in only one out of 56 (1·8%) patients during hospitalization [97]. Although elevation of liver enzymes is frequently transient in mild cases of the disease, significant elevation of liver enzymes is observed in severe COVID-19. Liver injury associated with COVID-19 is not correlated to the risk of death; however, increased time of hospitalization has been observed in individuals who had raised liver enzymes [95].

Despite the highly expressed ACE 2 receptors on the biliary ducts, ALP was not found to be elevated in the majority of COVID-19 cases. The mechanisms leading to hepatic injury in COVID-19 is multifactorial and could be the result of direct invasion of the virus via the biliary ducts, pneumonia-associated hypoxia, CRS and drug-induced liver injury (DILI) related to lopinavir/ritonavir. Biopsy analysis of three patients infected with SARS-CoV suggests direct viral invasion of the virus to the hepatocytes [98]. Limited information exists on the infectivity of SARS-CoV-2 in the liver [99]. In post-mortem biopsy analysis of a liver from one COVID-19 infected patient, DILI, or viral damage could not be specified [50]. SARS-CoV is known to ameliorate liver injury in hepatitis B/hepatitis C infected patients; regarding COVID-19 the fatality rate and severity of illness in patients with underlying hepatic disease, and outcomes of co-infection of viral hepatitis are unclear [99].

Concomitant kidney and liver injury in severe COVID-19 may result in decreased metabolism of medications and increased risk of drug toxicity [100]. To avoid further complications in severe COVID-19, clinicians should be aware of the precautions on the use of medications with potential hepatotoxicity, monitor side effects and consider the required drug dose adjustment.

### Endocrine involvement

Observational studies indicate that COVID-19 is associated with an increased risk of diabetic ketoacidosis and hyperglycemia. Dysregulation of ACE 2 pathways may cause alterations in glucose metabolism [101,102]. Pancreatic cells, including both the islet cells and exocrine cells, express a considerable amount of ACE 2 receptors. Clinical findings of mild pancreatic injury have been observed in 1–2% and 17% of mild and severe COVID-19, respectively. Liu *et al.* postulated the possible involvement of the pancreatic tissue in COVID-19 based on these clinical findings. In patients with severe disease, parenchymal inflammation of the pancreas results in the accumulation of immune system cells, particularly neutrophils and macrophages. Subsequent cytokine production and migration of macrophages may deteriorate lung injury and accelerate the processes leading to ARDS [103].

The results of a retrospective cohort in Hamburg, Germany demonstrated that 68% of the critically ill male COVID-19 patients suffer from low levels of testosterone and dihydrotestosterone. They also found that elevated levels of estradiol in males correlate with IL-6 levels. On the contrary, in females, a positive association was found between testosterone levels and IL-6 [104]. As previously mentioned, the Leydig cells could be a potential target for SARS-CoV-2. Another explanation for disturbances observed in sexual hormones could be the CRS [17].

### Obstetric & gynecologic complications

Regarding the risk of intrauterine transmission of COVID-19 uncertainties exist. Limited evidence suggests that vertical transmission of COVID-19 during late pregnancy is possible [105]. Increased oxygen demand and physiologic anemia during pregnancy are the potential factors that could exacerbate the severity of COVID-19. Besides, the attenuation of Th1 response and stimulation of Th2 environment is contributed to susceptibility to viral infections [30]. Data on the clinical implications of COVID-19 in pregnancy is limited to case reports and case series. According to a review of the case series, among the 32 pregnant women infected with SARS-CoV-2, 6% required ICU care. In 47% of the patients, preterm delivery occurred; one woman had a stillbirth and, one delivery resulted in neonatal death [106]. COVID-19 probably increases the risk of miscarriage and intrauterine growth restriction [107]. In an observational cohort study on 42 pregnant women, signs and symptoms imitating preeclampsia (hypertension, proteinuria, elevated liver enzymes and thrombocytopenia) were observed in 14% of the pregnant women infected with SARS-CoV-2 [108]. The underlying etiologies of these findings in pregnant women are not completely understood and warrants further investigation.

### GI tract involvement

GI symptoms infrequently accompany COVID-19 pneumonia. About 2–10% of patients with COVID-19 had GI symptoms such as diarrhea, abdominal pain and vomiting [109]. Interestingly, diarrhea could be one of the initial presentations of the disease. According to Parasa *et al.* systematic review and meta-analysis on 23 published and six preprint studies with a total of 4805 patients, the incidence rate of diarrhea and nausea or vomiting is 7.4% (95% CI: 4.3–12.2%), and 4.6% (95% CI: 2.6–8.0%), respectively [94].

Epithelial cells of the GI tract are enriched with ACE 2 receptors and SARS-CoV-2 RNA has been detected in stool specimens of the infected patients [3]. Based on data from biopsy analysis, direct viral invasion can cause GI symptoms in COVID-19 patients [110]. ACE 2 plays a fundamental role as an anti-inflammatory enzyme of the GI tract. Disturbance in the RAS system may result in diarrhea associated with COVID-19 [111]. These findings, along with the fact that the virus can be viable within fecal excretion for some time, suggest that COVID-19 could also be transmitted via the fecal-oral route.

### Neuromuscular involvement

In a retrospective study from a local hospital in Wuhan, different neurologic manifestations suggestive of the central nervous system (CNS), peripheral nervous system (PNS) and musculoskeletal involvement were reported. These symptoms occurred in 36% of the infected patients [112]. CNS symptoms (24%) presented as dizziness, headache, impaired consciousness, cerebrovascular disease, ataxia and epilepsy. In a small number of patients (2–10%), hypogeusia, hyposmia and neuralgia were detected [112]. Epithelial cells of the nasal and oral cavity are enriched with ACE 2 receptors. It is postulated that SARS-CoV-2 could enter the CNS via the olfactory bulb and impair the function of sensory neurons. Post-infectious hypogeusia and hyposmia associated with COVID-19 are more frequently observed in younger patients and in females [113].

In the study conducted by Mao *et al.* who investigated the neurological manifestations of the COVID-19 skeletal muscle injury was detected in 19% of the patients with severe infection. Lactate dehydrogenase (LDH) and creatine phosphokinase (CPK) elevations consistent with muscular injury could be implicative of the possible invasion of the virus into the peripheral nerves and muscles [112]. Interestingly in a few reports, rhabdomyolysis associated with SARS-CoV-2 infection has been described [114,115]. In one of the cases the CPK level raised to 42,000 U/l [115]. The pathophysiology of rhabdomyolysis in COVID-19 is poorly understood; some experts believe that the virus could invade the myocytes through ACE 2 receptors [112]. Other explanations such as toxin-induced injury, deposition of the virus antibody complexes and T-cell mediated injury have also been suggested [115].

In a few reports, acute disseminated encephalomyelitis (ADEM) linked to COVID-19 has been described. These cases presented with neurologic symptoms including dysphagia, dysarthria, aphasia and coma weeks after the initial infection. Consistent with ADEM, magnetic resonance imaging (MRI) demonstrated hyperintensities in the white matter and oligoclonal bands were present in cerebrospinal fluid (CSF) analysis [116]. ADEM appears to be caused by an autoimmune inflammatory reaction triggered by SARS-CoV-2 in genetically predisposed patients [117]. Observations from case series and case reports indicate that Guillain Barre syndrome is another neurologic complication proceeded by COVID-19. Progressive weakness of extremities, paresthesia, facial diplegia, ataxia, and bulbar weakness occurred 5–14 days after the infection. However, antiganglioside antibodies were not found in CSF analysis. Electrophysiological findings were consistent with axonal and demyelinating neuropathy [118,119].

### Central nervous system involvement

More than three-fourth (88%) of the patients with severe COVID-19 displayed neurologic manifestations, including acute cerebrovascular diseases and encephalopathy. Interestingly, in patients with CNS involvement, the disease was more severe, and lymphopenia, elevated ferritin and LDH levels were noteworthy [112]. Neuroinvasive feature of the betacoronaviruses and the presence of SARS-CoV in the CNS has been confirmed in the previous studies. Because of the structural and pathogenic similarities to SARS-CoV (ACE 2-mediated entry), acute respiratory and cardiovascular failure of COVID-19 has been linked to the presumptive neuroinvasive potential of SARS-CoV-2 [120]. The virus is believed to enter the CNS via the systemic circulation in the case of severe infection. Another possible route of entry could be from the cribriform plate through the retrograde neuronal pathway, which is a possible explanation for hyposmia [121]. Besides, some viruses belong to the Coronaviridae family have been demonstrated to spread via a synapse-connected route to the medullary cardiorespiratory center from both the mechanoreceptors and chemoreceptors in the lungs as well as lower respiratory airways [120].

Acute ischemic stroke is recognized as a neurologic complication of COVID-19 particularly in elderly, hypertensive and atrial fibrillation patients; although it could occur even in young patients with no risk factors [122]. Increasing evidence suggests that SARS-CoV-2 stimulates a prothrombotic environment which induces endothelial cell activation, tissue factor expression, thrombin production and hypercoagulability. Large-vessel occlusion has been found to occur with elevated D-dimer levels (≥1000μg/l) [123]. Furthermore, the presence of antiphospholipid antibodies could increase the risk of cerebral infarcts [91].

On 4 March 2020, the first isolation of the virus genome from the cerebrospinal fluid of a patient with confirmed COVID-19 at Beijing Ditan Hospital, China, was reported [124]. In a recent report, a presumptive case of necrotizing encephalopathy associated with COVID-19 was described. The patient's symptoms included fever, cough and impaired mental status. SARS-CoV-2 was detected in the nasopharyngeal swab. CSF bacterial culture and tests for the possible viruses were negative. Unfortunately, the test for SARS-CoV-2 could not be performed. Virus-induced intracranial CRS and possible blood–brain barrier damage may have caused hemorrhagic encephalopathy [125]. In another report, SARS-CoV-2 was detected in CSF analysis of an 11-year-old child who presented with status epilepticus and was later diagnosed with COVID-19-associated encephalitis. Invasion of the virus via ACE-2 receptors may cause injury of the vascular endothelium [126].

### Ocular involvement

SARS-CoV has been detected from the tear samples in the previous reports. Evidence suggests possible conjunctivitis related to SARS-CoV via inoculation of droplets to the eyes, lacrimal infection and virus migration from the nasolacrimal duct [127]. Conjunctival hyperemia and eyelid edema have been reported as initial manifestations of COVID-19. Anecdotal evidence indicates that 2–32% of the COVID-19 cases experience ocular symptoms [128]. Ocular manifestations of COVID-19 were investigated in a case series in Hubei province, China. Approximately, a third of the 38 cases presented with ocular symptoms including conjunctival hyperemia, chemosis, epiphora and increased secretions [129]. Of note, conjunctival swabs were positive for SARS-CoV-2 in 16% of the patients with ocular symptoms. Interestingly, leukocytosis, LDH, procalcitonin and C-reactive protein (CRP) levels were considerable in patients with ocular symptoms [129].

### Skin involvement

According to the present literature, cutaneous changes due to COVID-19 infection are infrequently observed. Several skin conditions, including erythema, papules, maceration and scaling accompanied with symptoms of burning, itching and stinging, are mostly related to personal protective equipment and personal hygiene measures [130]. Recently, a report of skin rash with petechiae was described as a possible early sign of COVID-19 in Thailand [131]. Later, Recalcati in the Lecco Hospital, Lombardy, Italy reported skin manifestations in 18 out of 88 (20.4%) COVID-19 patients. These manifestations either existed at the time of admission or developed during the hospital stay. Cutaneous involvements included erythematous rash (77.78%), widespread urticaria (16.67%) and chickenpox-like vesicles (5.56%). These skin lesions were either along with mild itching or pruritus was absent. The possible correlation between skin involvement and severity of COVID-19 was not observed [132]. Table 1 summarizes organ/system complications with related signs/symptoms, laboratory abnormalities and pathogenic mechanisms in patients with COVID-19. Clinical complications of COVID-19 are also schematically shown in Figure 1.

**Table 1.** Clinical manifestations, laboratory abnormalities and risk factors contributed to organ involvement in COVID-19.

Organ involvement associated with COVID-19	Clinical manifestations/signs and symptoms	Associated laboratory abnormalities	Risk factors	Pathogenic mechanisms	Ref.
Respiratory system	Mild (fever, cough, fatigue, anorexia, dyspnea, myalgia, sore throat, nasal congestion, headache, diarrhea, nausea, vomiting, hyposmia)	Increased hs-CRP lymphocytopenia, prolonged PT, elevated LDH	–	Direct viral invasion	[32,39,50]
	Moderate pneumonia (fever, cough, dyspnea, tachycardia, blood oxygen saturation levels (SpO_2_) ≥90%)	Increased hs-CRP lymphocytopenia, prolonged PT, elevated LDH	Males > females	Direct viral invasion	[32,39,42,50,51]
	Severe pneumonia (fever, cough, dyspnea, tachycardia, blood oxygen saturation levels [SpO_2_] <90%)	Neutrophilia, elevated LDH and D-dimer, elevated hs-troponin I lymphocytopenia Increased hs-CRP	Males > females Elderly DM HTN Age Malignancy, CeVD, CKD	Direct viral invasion; virus-induced pancreatitis; respiratory failure due to hypokalemia and hypophosphatemia; respiratory failure due to neuroinvasive potential of the virus; ACE 2 downregulation; CRS	[27,32,39,42,50,51, 56,63,92,103, 120,137]
Cardiovascular system	ACS (newly discovered EKG abnormalities)	hs-troponin T elevation, higher leukocyte counts, lower lymphocyte counts, higher levels of D-dimer, CRP, procalcitonin, NT-proBNP	Elderly, males > females HTN, CAD, CKD, CHF	Insufficient cardiovascular reserve and inflammatory response; plaque destabilization; hypoxia induced by ARDS	[39,59]
	Malignant arrhythmia and exacerbation of heart failure	hs-troponin T and NTproBNP elevation	CHF, CAD	Insufficient cardiovascular reserve and inflammatory response; hypokalemia	[56,59,67]
	Fulminant cardiomyopathy (cardiogenic shock)	–	Pregnancy (case report); African–American ethnicity (case report); morbid obesity (case report)	High inflammatory burden and CRS; possible neuroinvasive potential	[59,61–63,67, 121,137]
	Pericardial effusion and cardiac tamponade	–	No identified risk factors	High inflammatory burden and CRS	[66,67,137]
Kidneys	AKI (proteinuria, hematuria)	Elevation of BUN and SrCr; CPK; abnormal urine analysis (microalbumin,α1-microglobulin, immunoglobulin-G and transferrin)	Elderly, HTN, CHF, DM	Direct viral invasion; deposition of immune complexes; CRS; hypoxia, shock; rhabdomyolysis; nephrotoxins	[44,46,70,72,73, 76,137]
	Electrolyte imbalance	Hypokalemia		Disturbance in ACE 2/Ang 1–7 axis	[20,56]
Endocrine involvement	Mild pancreatitis	Amylase and lipase evelation		Direct viral invasion (?)	[103]
	Diabetic ketoacidosis, hyperosmalarity	Hyperglycemia	Diabetes mellitus	Disturbance in ACE 2/Ang 1–7 axis	[101,102]
Obstetric complications	Preterm birth, Intrauterine growth restriction, miscarriage, preeclampsia-like syndrome	Hypertension, proteinuria, elevated liver enzymes, thrombocytopenia	–	Vasoconstriction because of renin-angiotensin disturbance	[30,106–108]
Blood cells	Thrombocytopenia	–	–	Direct viral invasion; CRS; Alveolar damage affect the resident megakaryocytes; thrombosis formation	[79–81,137]
	Decreased hemoglobin	–	–	Viral proteins bind to porphyrin	[23]
Immune system	Lymphopenia, macrophage damage, decreased CD8^+^ T cells, decreased NK cells, T-cell exhaustion	Elevation of TNF-α, IL-6 and IL-10	–	Direct viral invasion to CD169^+^ macrophages IL-6-induced lymphocyte apoptosis	[24,25,32,82]
Liver	Mostly asymptomatic	Elevation of ALT, AST, γ-GT, LDH, and bilirubin (rare)	Males > females adults severe disease	DILI, SIRS CRS Hypoxia Possible direct viral invasion (?) Possible role of metabolites entering through gut–brain axis(?)	[95,97,137]
Gastrointestinal system	Diarrhea, abdominal pain, nausea, vomiting, anorexia	Not identified		Direct viral invasion	[95]
Coagulation dysfunction	SIC and DIC; large-vessel stroke; APS; VTE	Elevation of D-dimer and FDP levels, PT and thrombocytopenia	Severe disease	Hypoxia-induced coagulation dysfunction Direct viral invasion (to endothelial cells) Immobility	[83–86,91,122]
Central nervous system	Dizziness, fatigue, headache, impaired consciousness, Ischemic stroke, ataxia, epilepsy; necrotizing encephalopathy; cerebral hemorrhage	Thrombocytopenia, higher BUN, lymphocytopenia	Severe disease > nonsevere disease Lower lymphocyte count (probable immunosuppression)	Possible role of the metabolites entering through the gut–brain axis (dizziness and fatigue); direct viral injury via respiratory droplets or hematogenous route; possible intracranial CRS (encephalopathy)	[112,121,125]
Peripheral nervous system	Hypogeusia, hyposmia, neuralgia	–	Female patients, younger patients	Possible direct viral injury	[112,113]
	Guillain-Barre;	–	–	Autoimmune inflammatory reaction triggered by the virus	[118,119]
	ADEM	–	–	Autoimmune inflammatory reaction triggered by the virus	[117]
Musculoskeletal	Myalgia, rhabdomyolysis	Neutrophilia, lymphocytopenia, increased CRP and D-dimer, In severe disease: increased ALT and AST, SrCr, CPK, LDH	No identified risk factor	Possible direct viral injury; hypokalemia, viral toxin, T-cell-mediated response, deposition of the virus antibody complex	[75,112,115]
Skin involvement	Erythematous rash, widespread urticaria, chickenpox-like vesicles, petechiae	–	–	–	[131,132]
Ocular involvement	Conjunctival hyperemia, chemosis, epiphora and increased secretions	leukocytosis, LDH, procalcitonin and CRP levels	–	Possible lacrimal infection and virus migration from the nasolacrimal duct	[127–129]
PIMS-TS	Unrelenting fever, rash, nonpurulent conjunctivitis, edema, nausea, abdominal pain, myalgia, odynophagia, pericardial effusion, ascitic effusion, severe gastrointestinal symptoms, myocarditis, coronary artery abnormalities, TSS	Leukopenia, Thrombocytopenia Elevation of IL-6, procalcitonin, C-reactive protein, ferritin and D-dimer; Hypoalbuminemia	African ancestry	CRS, antibody-dependent enhancement	[141,143]
Multiorgan failure in adults	Septic shock, AKI, cardiac injury, ARDS, liver failure	Lymphocytopenia, thrombocytopenia, ↑Ferritin, ↑D-dimer, ↑PT, ↑FDP, ↑CRP, myoglobin, ↑IL-6, ↑NLR, ↑PLR	Immunosuppressed patients	CRS, sHLH	[79,133,136,137]

ACS: Acute coronary syndrome; ADEM: Acute disseminated encephalomyelitis; ALT: Alanine transaminase; ARDS: Acute respiratory distress syndrome; AST: Aspartate aminotransferase; CAD: Coronary artery disease; CeVD: Cerebrovascular disease; CHF: Chronic heart failure; CKD: Chronic kidney disease, CLD: Chronic liver disease; CPK: Creatine phosphokinase; CRP: C-reactive protein; CRS: Cytokine release syndrome; CVD: Cardiovascular disease; DIC: Disseminated intravascular coagulation; DILI; Drug-induced liver injury; FDP: Fibrin degradation products; γ-GT: Gamma-glutamyl transferase; HIV: Human immunodeficiency virus; HTN: Hypertension; IL-6: Interleukin 6; LDH: Lactate dehydrogenase; NLR: Neutrophil/lymphocyte ratio; PIMS-TS: Pediatric inflammatory multisystem syndrome temporally associated with SARS-COV-2; PLR: Platelet/lymphocyte ratio; PT: Prothrombin time, SIC: Sepsis-induced coagulopathy; SIRS: Systemic inflammatory response; sHLH: Secondary haemophagocytic lymphohistiocytosis; TSS: Toxic shock syndrome.

**Figure 1.** The clinical complications of COVID-19. ACE 2: Angiotensin-converting enzyme 2; ACS: Acute coronary syndrome; ADEM: Acute disseminated encephalomyelitis; Ang 1–7: Angiotensin 1–7; ARDS: Acute respiratory distress syndrome; BBB: Blood–brain barrier; DILI: Drug-induced liver injury; FDP: Fibrin degradation products; NK cell: Natural killer cell.

### Multiorgan failure

After the internalization, SARS-CoV-2 replicates over a few days, and the innate immunity fails to combat the virus. In this phase, relatively mild symptoms are observed. If the adaptive immune system succeeds in decreasing the viral load, convalescence is expected; meanwhile, in some patients, CRS induces dysregulated immune response causing further tissue damage [133]. A multi-center observational study on 109 decedents with COVID-19 pneumonia from three hospitals in Wuhan, China, demonstrated that multiple organ failure, especially respiratory failure and heart failure, occurred in near all patients even at the early stage of the disease. The mean ± standard deviation time onset from early symptoms to death in the cohort was 22.3 ± 9.2 days [134]. On the other side of the world in France, Lescure *et al.* described five patients as the first cases of COVID-19 in Europe. One of these cases was an 80-year-old man who presented with diarrhea and fever. His symptoms rapidly progressed toward ARDS, AKI, liver failure and shock. The patient received broad-spectrum antibiotics and remdesivir; however, he died at day 24 of illness [135].

The pathogenesis of multiorgan dysfunction in COVID-19 has been contributed to secondary hemophagocytic lymphohistiocytosis (sHLH), an overreactivated and dysregulated immune response triggered by viral overload, which results in CRS and deterioration of the disease. Resembling 50% of critical cases of COVID-19, cytokine elevation, cytopenia, fever and high ferritin levels are the distinct features of HLH [136,137]. Evidence for the role of corticosteroids to suppress the hyperstimulated immune response is limited; therefore, the Surviving Sepsis Campaign (SSC) guidelines published in March 2020 does not make any recommendations on their clinical use [138].

### Kawasaki-like syndrome

The first case of Kawasaki-like syndrome associated with COVID-19 was a 6-month-old infant who presented with fever, fussiness, maculopapular rash, conjunctivitis, swelling of the extremities and tongue papilla. The result of RT-PCR was positive for COVID-19. These symptoms occurred 3 weeks after her probable exposure to SARS-CoV-2 [139]. Subsequently, when clusters of children presenting with Kawasaki-like symptoms were admitted in hospitals in Italy and France, concerns over COVID-19 in the pediatric population raised [140,141]. Kawasaki disease linked to COVID-19 was named Pediatric Inflammatory Multisystem Syndrome Temporally associated with SARS-CoV-2 (PIMS-TS) and Multisystem Inflammatory Syndrome in children (MIS-C). This hyperinflammatory syndrome presents 2–4 weeks after infection and manifests as unrelenting fever, rash, nonpurulent conjunctivitis, edema, nausea, abdominal pain, myalgia, odynophagia and pericardial effusion [142]. A considerable number of PIMS-TS cases are complicated with severe gastrointestinal symptoms, myocarditis, coronary artery abnormalities and toxic shock syndrome (TSS). Most children presenting with PIMS-TS fulfilled the criteria of macrophage activation syndrome (MAS) in the study conducted by Verdoni *et al.* Leukopenia, thrombocytopenia and elevation of the biomarkers of inflammation (IL-6, procalcitonin, CRP, ferritin and D-dimer) and, hypoalbuminemia are frequently reported in children presenting with PIMS-TS. The possible link to the antibody-dependent enhancement and hyperstimulated cytokine release are presumed to be responsible for PIMS-TS [143]. Genetically predisposed children particularly those of African ancestry are probably at greater risk of COVID-19-associated Kawasaki [141]. Anti-inflammatory agents particularly high-dose IVIG and methylprednisolone are probably beneficial treatments for PIMS-TS [142,143].

## Conclusion & future perspective

This review tried to discuss the current literature on the complications of COVID-19, the prognostic value of laboratory abnormalities, histopathologic evidence of virus invasion and expert comments on the pathogenesis of the disease. Respiratory system and the lungs are the most commonly involved sites of COVID-19 infection. Therefore, pulmonary signs and symptoms are generally early onset, more prominent and, relatively well described. Apart from the pulmonary system, other organs/systems, including cardiovascular, liver, kidneys, gastrointestinal and central nervous systems are involved with different frequencies and degrees of severity. On the other hand, mucocutaneous, and endocrine complications of COVID-19 are quite uncommon based on the current literature. The major electrolyte imbalance that may be involved in either the development or worsening of ARDS and acute cardiac injury in the setting of COVID-19 is hypokalemia. As far as we know, ARDS, AKI and myocardial infarction are associated with worse outcomes of COVID-19. Elevation of inflammatory biomarkers (CRP, ferritin, neutrophil/lymphocyte ratio, platelet/lymphocyte ratio), lactate dehydrogenase, hypokalemia, hypophosphatemia and coagulopathy (elevated D-dimer and PT, hypofibrinogenemia) reflect the progression of the disease and are predictors of death.

Regarding the virulence and pathogenesis of SARS-CoV-2, direct viral invasion and damage to targeted tissue have been proposed. However, some questions remain unanswered. Expression of ACE 2 receptors is considerably higher in the GI tract, kidneys, testis and heart than in the lungs; meanwhile, there is no positive correlation between the level of ACE 2 expression and SARS-CoV-2 tissue tropism. Whether ACE 2 is the only receptor related to the infectivity of SARS-CoV-2 requires further to be studied. Furthermore, it is not elucidated if cells enriched with ACE 2 receptors (such as cholangiocytes, Leydig cells, and cells in seminiferous ducts of testis) or organs at risk of exposure to the virus (the eyes), are targeted. Another issue is the concerns over SARS-CoV-2 because of its potential ability of mutation. Epidemiologic and genomic investigations are required to predict how the viral mutations and ACE 2 polymorphism will affect the pathogenesis and invasion of the virus. The possible beneficial or detrimental functions of ACEIs and ARBs on the course of disease and outcome are other questions that remain to be answered in this regard. Although COVID-19 is not a metabolic disease, several studies indicate the link of the ACE 2/angiotensin system and pathogenicity of the disease. To improve the survival rate and disease severity, management of blood pressure and blood glucose is highly recommended. ACE 2/angiotensin system seems to play a fundamental role in the inflammatory response and tissue injury of COVID-19. Apart from direct tissue invasion, impaired oxygenation and immune dysregulation (such as reduction of lymphocytic T cells and NK cells) also play roles in the pathogenesis of COVID-19 infection.

Secondary HLH and PIMS-TS are suggested to be the significant culprits of multiorgan failure (mostly ARDS and cardiomyopathy in secondary HLH; cardiovascular involvement in PIMS-TS), and consequently, death in cases of severe COVID-19 infection. On the other hand, COVID-19 appears to have also immunosuppressive effects through exhausting and decreasing T lymphocytes via interacting with inhibitory receptors on the surface of NK and T cells (such as NKG2A, PD-1 and TIM-3). Hence, immunomodulators with both anti-inflammatory and immunostimulant activities may be useful in attenuating disease severity, preventing multiorgan failure and death.

**Executive summary**

**Background**

- COVID-19 global pandemic is considered a public health emergency of international concern (PHEIC), as declared by the WHO.

**Objectives**

- Understanding the pathologic process of the disease provides us new insights into effective therapeutic approaches.

**Methods**

- A literature search in Pubmed, Scopus and Google Scholar for the relevant articles regarding clinical complications and pathogenesis of COVID-19 was conducted.

**Results**

- Related articles were included and discussed in this review.

**Conclusion**

- Respiratory system and the lungs are the most commonly involved sites of COVID-19 infection. Cardiovascular, liver, kidneys, gastrointestinal and central nervous systems are involved with different frequencies and degrees of severity.
